The article "Clinical Research of Combined Arteriovenous Approach Embolization on Complex Carotid-Cavernous Fistulas" was retracted in 2024. Reasons: signs of a paper mill; suspected computer-generated content; unreliable results or conclusions; concerns about the data.

# Clinical Research of Combined Arteriovenous Approach Embolization on Complex Carotid-Cavernous Fistulas

**DOI:** 10.1155/2021/5580957

**Published:** 2021-05-27

**Authors:** Li Xinxing, Zheng Jihui

**Affiliations:** ^1^Department of Neurosurgery, Shengjing Hospital of China Medical University, Shenyang, 110004 Liaoning, China; ^2^Department of Radiology, The Fourth Affiliated Hospital of China Medical University, Shenyang, 110032 Liaoning, China

## Abstract

The objective of this study was to observe the curative effect of combined arteriovenous approach embolization on complex carotid-cavernous fistulas. The clinical data of 13 patients with complex carotid-cavernous fistulas treated with combined arteriovenous approach embolization in our department between January 2017 and January 2020 were analyzed retrospectively. All 13 patients received the combined arteriovenous approach embolization with coil combined with Onyx glue. The intraoperative angiography immediately showed that the fistula could be completely blocked, and the carotid artery was/got unobstructed. The patients had no clinical symptoms recurring during a follow-up period of 3-18 months, on average 9.1 ± 6.3 months. A combined arteriovenous approach embolization on complex carotid-cavernous fistulas is safe and effective since it can improve the occlusion rate and reduce the relapse rate.

## 1. Introduction

In recent years, as the development of intervention materials and technologies progressed, most traumatic carotid-cavernous fistulas (TCCF) can be embolized and the fistulas can be occluded via technologies like artery approach application or combined application of coil, liquid embolic agents (NBCA or Onyx glue), and endovascular covered stent [1, 2]. But for some complex CCF, if the fistulas are too big or too small and the fracture sites or fistulas are angulated with blood vessels, the artery pathway cannot reach or completely block the fistulas. This will lead to the vestigial and relapse of fistulas, and sometimes, the internal carotid artery (ICA) will be sacrificed [3]. Combined arteriovenous approach using coil and liquid embolic agent- (NBCA or Onyx glue) assisted technologies occludes fistulas and improves the cure rate of CCF. This study retrospectively analyzes the clinical data of 13 patients with complex carotid-cavernous fistulas treated with combined arteriovenous approach embolization of coil combined with Onyx glue. The report is as follows.

## 2. Materials and Methods

### 2.1. General Data

13 patients diagnosed and treated at Shengjing Hospital of China Medical University from January 2017 to January 2020 were collected. Among them, 9 cases were male and 4 cases were female, aged 31-68 years (45.9 ± 8.3). All of them are traumatic. Before the treatment, all of the 13 patients were seen with varying degrees of intracranial murmur and bulbar conjunctival congestion edema accompanied by pulsating exophthalmos, among which 11 cases were unilateral and 2 cases were bilateral. Ten cases showed ocular motility disorders, while five cases showed impaired vision. According to Barrow's CCF typing from 1985, the following types are discussed: (1) Type A—the ICA is directly communicated with cavernous sinus; (2) Type B—the ICA is communicated with cavernous sinus through rami meningeus; (3) Type C—the rami meningeus of external carotid artery is communicated with cavernous sinus; and (4) Type D—both internal carotid and external carotid are communicated with cavernous sinus through their own rami meningeus, respectively [4]. All these 13 patients are Type D (Figures 1(a)–1(d)) and treated with endovascular treatment.

The exclusion criteria were as follows: (1) patients suffering from heart, lung, liver, kidney, and other severe diseases and who are thus unable to get operated; (2) coagulation disorders; (3) patients who are allergic to meglumine diatrizoate who are unable to undergo operation; and (4) family members of patients who did not sign the informed consent.

This research was approved by the Ethics Committee of the Shengjing Hospital of China Medical University. All family members of the patients had signed the informed consent.

### 2.2. Therapeutic Methods

After successful anesthesia, bilateral punctures were used. An 8F artery sheath catheter was inserted in the right-side femoral artery, and a 6F artery sheath catheter was inserted in the left-side femoral vein. A 6F long sheath was placed in the petrous carotid artery using coaxial technology. An anteroposterior and lateral film and 3D rotation angiography were conducted via a long sheath. Choosing the right operating angle, the location and diameter of the fistula were measured. Under the guidance of intravenous roadmap, a long sheath was guided into the petrous carotid artery in reserve. A 6F Guiding catheter was placed in jugular bulb using coaxial technology. Under the guidance of intravenous roadmap, a micro-wire and Echelon-10 microcatheter were placed in the front of the affected side cavernous fistula through inferior petrosal sinus. After the Echelon-10 microcatheter was entered into the cavernous fistula, microcatheter angiography was conducted to measure the location of fistula and the size of cavernous fistula and choose the right coil blocking the cavernous fistula. After blood-flow decrease was confirmed via internal carotid angiography, with Echelon-10 microcatheter angiography, Onyx glue was slowly injected in low doses according to blood flow velocity of the fistula to assist embolization. In some cases, the hyperglide balloon was used through artery approach and occluded the fistula to stop Onyx glue from flowing backwards to carotid artery through the fistula. To identify the closure of fistula, internal carotid angiography could be conducted discontinuously during the process of slow injection of Onyx glue to confirm the fistula was completely blocked.

### 2.3. Follow-Up

During a follow-up period of 3-18 months (average of 9.1 ± 6.3 months), the clinical symptom improvement or severity of patients was recorded. Moreover, CTA or MRA was reexamined to observe if patients' pulsating exophthalmos, intracranial murmur, and bulbar conjunctival congestion edema have disappeared or have been relieved.

## 3. Results

All 13 patients were treated with artery approach combined with transvenous approach through inferior petrosal sinus (Figures 2(a)–2(c)). Microcatheters were all successfully placed on the cavernous sinuses through inferior petrosal sinuses, and Onyx glue combined with coil was used to embolize. Intraoperative angiography immediately showed that the fistula was completely blocked, and the internal carotid artery was unobstructed and uninfluenced (Figures 3(a)–3(d)). After the treatment, the intracranial murmur and pulsating exophthalmos in 13 patients have all disappeared, and the bulbar conjunctival congestion edemas completely disappeared postoperatively within 1-8 weeks (Table 1). Out of 10 patients with ocular motility disorders, 9 patients recovered after 2-3 weeks, 1 patient did not recovered, and there is no new oculomotor nerve palsy. In 5 patients with impaired vision, the vision of 3 patients was improved, and the impaired vision of 2 patients had no obvious remission, only with light perception. One patient had new abducens nerve palsy, and the symptoms were gradually relieved and finally disappeared within 3 months. After the operation, 7 patients had varying degrees of headache and nausea, but all were relieved within 2 weeks. All of the 13 cases had no internal carotid artery occlusion, distal cerebral infarction, or cerebral hemorrhage symptoms. All of the 13 patients had no clinical symptoms recurrence during a follow-up period of 3-18 months (average of 9.1 ± 6.3 months). Reexamining CTA and MRA, patients had no internal carotid artery occlusion, distal cerebral infarction, or cerebral hemorrhage. Figures 3(e)–3(g) show the ocular features of one of the patients before and after surgery. It can be clearly seen that the patient recovered normally at 3 months after surgery without bulbar conjunctival congestion and protrusion of the eye.

## 4. Discussion

TCCF are mostly caused by skull base fractures in the middle cranial fossa, which leads to the tear of the cavernous segment of the internal carotid artery or its branches and the short circuit between the internal carotid and the cavernous sinus. Arterial blood flows into the cavernous sinus via laceration, which makes branches of veins around the cavernous sinus (e.g., superior ophthalmic vein) refluent and expand. This leads to pulsating exophthalmos, bulbar conjunctival congestion edema, and intracranial murmur [5, 6]. The purpose of TCCF treatment is to protect vison and eliminate intracranial murmur. The ideal therapy is to block the fistula and keep the internal carotid unobstructed at the same time [7]. At present, the therapies of TCCF mainly include artery approach embolization of detachable balloon, stent-graft embolization, and transvenous approach embolization of coil combined with liquid glue among others [8]. Low expense and simple operation are the advantages of detachable balloon treatment, which is the classical therapy of TCCF. But some patients may have cerebral infarction or TCCF recurrence because of balloon premature detachment or deflation. In some complex TCCF, the fistula is too small or at an angle with ICA, so the balloon cannot enter, or the fistula is so large that the balloon cannot completely block the fistula [9]. Stent-graft embolization is the major therapy of TCCF today. It applies to patients with tiny fistulas, especially those with TCCF combined pseudoaneurysm [10]. Stent-graft utilizes the biofilm on the stent surface to block the fistula directly and keep the carotid artery unobstructed. But due to stent-graft's poor flexibility, it is not suitable for tortuous blood vessels. It may be severely restricted to block collateral vessels playing important roles [11, 12]. As a result, for refractory TCCF, it has great significance to keep carotid artery unobstructed, and combined arteriovenous approach embolization is recommended.

Artery-inferior petrosal sinus combined approach embolization of coil combined liquid glue has gradually become the treatment of complex TCCF. It is mainly used for Type D TCCF patients according to Barrow's typing. Most other types of patients can be treated via arterial approach. If the fistula cannot be reached via the arterial approach, the combined arteriovenous approach can also be used. Type D TCCF patients have small fistulas, so microcatheters or balloons cannot pass [13]. Moreover, the location of fistulas is hard to deal with and the stability of microcatheters is poor. After detachable balloon embolization or coil embolization, patients with recurrent TCCF can also be treated with artery-inferior petrosal sinus combined approach embolization. Microcatheters enter into cavernous sinuses through inferior petrosal sinuses. With microcatheter angiography, the fistula of inferior petrosal sinus and the anatomic relationship of draining veins are carefully distinguished. The location of microcatheters is carefully adjusted, and appropriate coils are chosen to embolize. Relevant results of this study found that to make sure the fistula was completely blocked, cavernous sinus at the fistula needed to be embolized densely [14]. Just coil dense embolization may cause mass effect, which leads to cranial nerve palsy. In addition, more septation in cavernous sinus is easy to hinder the release of a coil, which leads to postoperative recurrence. Using coil dense embolization only cannot achieve a therapeutic effect. Therefore, loose embolization of coil combined with Onyx glue was used in this study. The results of this study revealed that loose embolization of coil can slow down the blood flow in cavernous sinus and reduce abnormal embolization of Onyx glue. Onyx glue has good controllability and can be injected slowly and discontinuously. Discontinuous injection changes the flow direction of Onyx glue. It can effectively fill the interspace left by loose embolization of coil. In the process of injection, arteriography was conducted many times to observe the effect of embolization.

Liquid glue's reflux to internal carotid via fistula is the most severe complication of TCCF treatment. It might be related to fast speed of injecting glue [15]. If blood flow velocity of the fistula is fast, injecting fast can easily cause Onyx glue to reflux to internal carotid, which will lead to an ischemia stroke [16]. Loose implantation of some coils in cavernous sinus slows down the blood flow velocity of the fistula. Meanwhile, slow and discontinuous injection of Onyx glue in low doses can reduce Onyx glue's reflux to internal carotid. In this study, however, these complications did not occur in all 13 patients. Some patients with big fistulas needed to use a hyperglide balloon via artery approach to occlude fistulas, which avoids Onyx glue's reflux to internal carotid. A combination of Onyx glue with coils was used for all 13 patients. The injection of DM-SO or Onyx glue in cavernous sinus may cause cranial nerve injuries in cavernous sinus, which leads to cranial nerve palsy. One patient in this group had short-term abducens nerve palsy after the operation, but the symptoms were relieved after hormonotherapy and neurotrophic treatment.

The results of this study show that for refractory TCCF, traditional balloon embolization had a high relapse rate, but the combined arteriovenous approach embolization of coil combined with Onyx glue was safe and effective. The treatment of coil combined with Onyx glue for intracranial complex TCCF can improve the occlusion rate and reduce relapse rates. But this study with a small number of patients and short follow-up period certainly has its limitations. A randomized controlled trial with multicenter, larger cohort and long-term perspective is needed to further confirm this study's results.

## Figures and Tables

**Figure 1:** The anteroposterior and lateral angiography of the internal and external carotid artery. (a) The anteroposterior angiography of internal carotid artery. (b) The lateral angiography of the internal carotid artery. In (a) and (b), superior ophthalmic vein drainage can be seen. (c) The anteroposterior angiography of external carotid artery. (d) The lateral angiography of the external carotid artery. In (c) and (d), blood supplies from the external carotid artery branches can be seen.

**Figure 2:** The angiography of the internal jugular vein and a microcatheter surgical site. (a) The angiography of the internal jugular vein, and the inferior petrosal sinus can be seen. (b) The angiography of a microcatheter; fast blood flow at the fistula can be seen. (c) The anteroposterior angiography of the external carotid artery after implanting coils through a microcatheter; the blood flow of contralateral cavernous sinus slowed down.

**Figure 3:** The postoperative anteroposterior and lateral angiography of the internal carotid artery and preoperative and postoperative comparison of two eyes. (a) The anteroposterior angiography of the internal carotid artery. (b) The lateral angiography of the internal carotid artery. In (a) and (b), the cavernous sinus had no images, and the fistula disappeared. (c, d) Coils and Onyx glue for embolization. (e) Bulbar conjunctival congestion in two eyes and exophthalmos before operation. (f) Bulbar conjunctival congestion in two eyes and exophthalmos were improved after operation. (g) The patient had recovered to a normal condition and was left with no bulbar conjunctival congestion and exophthalmos, 3 months after operation.

**Table 1:** Clinical data of 13 cases of CCF patients treated by combined arteriovenous approach.

Patients	Intracranial murmur and pulsating exophthalmos	Bulbar conjunctival congestion edemas	Ocular motility disorders		Impaired vision		Postoperative complications
	Postoperation	Postoperation	Preoperation	Postoperation	Preoperation	Postoperation	
1	Disappeared	1 w disappeared	Yes	1 w recovered	—	—	Headache and nausea, 2 w relieved
2	Disappeared	1 d disappeared	Yes	5 d recovered	Yes	Improved	Headache and nausea, 1 w relieved
3	Disappeared	2 d disappeared	—	—	—	—	Headache and nausea, 1 w relieved
4	Disappeared	2 w disappeared	Yes	3 d recovered	Yes	Improved	Headache and nausea, 1 w relieved
5	Disappeared	8 w disappeared	Yes	1 w recovered	—	—	No
6	Disappeared	2 w disappeared	Yes	1 w recovered	—	—	No
7	Disappeared	8 w disappeared	Yes	5 d recovered	—	—	No
8	Disappeared	2 w disappeared	—	—	—	—	Abducens nerve palsy, 3 m disappeared
9	Disappeared	2 w disappeared	Yes	No recovered	Yes	No improved	Headache and nausea, 2 w relieved
10	Disappeared	2 d disappeared	Yes	2 w recovered	Yes	No improved	Headache and nausea, 2 w relieved
11	Disappeared	2 w disappeared	—	—	—	—	No
12	Disappeared	1 w disappeared	Yes	1 w recovered	Yes	Improved	No
13	Disappeared	6 w disappeared	Yes	2 w recovered	—	—	Headache and nausea, 1 w relieved

## Data Availability

All data generated or analyzed during this study are included in this article.

## References

[1] Bailey C. R., Ray-Mazumder N., Sedighi Manesh R. (2017). Carotid cavernous fistula. *Journal of General Internal Medicine*.

[2] Ajhoun Y., El Khoyali A., Aissa I. (2019). Direct carotid-cavernous fistula: an atypical presentation. *Pan African Medical Journal*.

[3] Mouchtouris N., Lang M. J., Stefanelli A. (2020). Cavernous-carotid fistula presenting with intracerebral hemorrhage in the absence of ocular symptoms. *World Neurosurgery*.

[4] Han W., Kim J. H., Kang H. I., Kim D. R., Moon B. G., Kim J. S. (2019). Transvenous embolization of dural carotid cavernous fistula through the supraorbital vein. *Journal of Cerebrovascular and Endovascular Neurosurgery*.

[5] Amuluru K., Al-Mufti F., Gandhi C. D., Prestigiacomo C. J., Singh I. P. (2016). Direct carotid-cavernous fistula: a complication of, and treatment with, flow diversion. *Interventional Neuroradiology*.

[6] Briggs R. G., Bonney P. A., Algan O., Patel A. D., Sughrue M. E. (2019). Bilateral carotid-cavernous fistulas treated with partial embolization and radiosurgery. *Cureus*.

[7] Niu Y., Chen T., Tang J., Jiang Z. Y., Zhu G., Chen Z. (2020). Detachable balloon embolization as the preferred treatment option for traumatic carotid-cavernous sinus fistula?. *Interventional Neuroradiology*.

[8] Gomez-Paz S., Vergara-Garcia D., Robinson M., Kicielinski K. P., Thomas A. J., Ogilvy C. S. (2019). Coil embolization of a carotid-cavernous fistula through superior ophthalmic venous access via external jugular vein puncture approach. *World Neurosurgery*.

[9] Sur S., Menaker S. A., Alvarez C. (2020). Multimodal management of carotid-cavernous fistulas. *World Neurosurgery*.

[10] Lang M., Habboub G., Mullin J. P., Rasmussen P. A. (2017). A brief history of carotid-cavernous fistula. *Journal of Neurosurgery*.

[11] Cezar-Junior A. B., da Silva Viturino U. A., de Carvalho E. V., Faquini I. V., Almeida N. S., Azevedo-Filho H. R. C. (2019). Blister aneurysms of the internal carotid artery: surgical treatment and management outcome from a single center experience. *Clinical Neurology and Neurosurgery*.

[12] Abdel Wahab M. A., Farouk N., Saleh O. I. (2019). Early outcomes of traumatic femoral artery aneurysm (open repair versus endovascular treatment). *Annals of Vascular Surgery*.

[13] Ohshima T., Kawaguchi R., Miyachi S., Matsuo N. (2019). Traumatic carotid-cavernous fistula associated with persistent primitive trigeminal artery successfully treated using in-stent coil embolization. *World Neurosurgery*.

[14] Sanal B., Nas O. F., Korkmaz M., Erdogan C., Hakyemez B. (2018). Endovascular treatment in traumatic and spontaneous carotid cavernous fistulas: with different embolization agents and via various vascular routes. *Journal of Vascular and Interventional Neurology*.

[15] Shim H. S., Kang K. J., Choi H. J., Jeong Y. J., Byeon J. H. (2019). Delayed contralateral traumatic carotid cavernous fistula after craniomaxillofacial fractures. *Archives of Craniofacial Surgery*.

[16] Holland L. J., Mitchell Ranzcr K., Harrison J. D., Brauchli D., Wong Y., Sullivan T. J. (2019). Endovascular treatment of carotid-cavernous sinus fistulas: ophthalmic and visual outcomes. *Orbit*.

